The article "Serum Level of CEACAM1 in Patients with Nonsmall Cell Lung Cancer and Its Clinical Significance in Cancer Tissue" was retracted in 2023. Reasons: signs of a paper mill; suspected computer-generated content; unreliable results or conclusions; concerns about the data.

# Serum Level of CEACAM1 in Patients with Nonsmall Cell Lung Cancer and Its Clinical Significance in Cancer Tissue

**DOI:** 10.1155/2022/7948010

**Published:** 2022-04-12

**Authors:** Wenjun Liu

**Affiliations:** Department of Clinical Laboratory, Ruijin People's Hospital of Jiangxi Province, Ruijin 342500, Jiangxi, China

## Abstract

**Objective:**

To analyze the expression of CEACAM1 in serum of patients with nonsmall cell lung cancer (NSCLC) and to explore the correlation and clinical significance between the expression of CEACAM1 and pathological parameters of NSCLC tissue.

**Methods:**

A total of 100 patients with NSCLC who underwent tumor resection were screened. Another 100 healthy patients in physical examination department were selected as control group. Venous blood and cancer tissue samples were collected. The expression of CEACAM1, TGF-*β*, VEGF-A, and IL-8 was detected.

**Results:**

The results of various indicators in the lung cancer group were much higher than those in the healthy group; CEACAM1 was significantly positively correlated with TGF-*β* expression. The later the clinical stage and the higher the degree of differentiation of cancer tissue specimens, the more the expression of CEACAM1 in serum samples.

**Conclusions:**

The expression level of CEACAM1 in the serum of NSCLC patients is strongly correlated with TGF-*β*, VEGF-A, and IL-8, indicating that serum CEACAM1 and TGF-*β* levels can predict the occurrence, progression, and prognosis of lung cancer and provide a target for future targeted therapy of lung cancer.

## 1. Introduction

Lung cancer is one of the major diseases threatening the health of the global population [1]. It is the number one killer of men, and nonsmall cell lung cancer accounts for 80–85% of the total lung cancer [2]. Early lung cancer can choose neoadjuvant radiotherapy and chemotherapy combined surgical treatment and has a good therapeutic effect. [3] However, due to the long incubation period of lung cancer, the early symptoms are not obvious; most patients are diagnosed when lung cancer is advanced, and advanced lung cancer lost the chance of radical surgery due to malignant metastasis and was not sensitive to radiotherapy and chemotherapy [4, 5]. At present, the diagnosis of lung cancer mainly relies on the traditional bronchoscopy of central lung cancer and computerized tomography (CT) guided chest fine needle aspiration, combined with CT and PET imaging examination and serological lung cancer biomarker detection, etc. [6]. The detection of CA153, CA199, CA125, and AFP in many nonsmall cell lung cancer patients also has certain reference significance. How to improve the early detection efficiency of lung cancer and provide a greater chance of survival for lung cancer patients has become an urgent problem to be studied and solved.

The article "Serum Level of CEACAM1 in Patients with Nonsmall Cell Lung Cancer and Its Clinical Significance in Cancer Tissue" was retracted in 2023. Reasons: signs of a paper mill; suspected computer-generated content; unreliable results or conclusions; concerns about the data.

Carcinoembryonic antigen associated cell adhesion molecule 1 (CEACAM1) is a widely expressed immunoglobulin-like cell adhesion molecule that has a wide range of biological functions in regulating cell signaling [7]. Some studies have examined the expression of CEACAM1 in prostate cancer and found that it can be used as an indicator for early diagnosis of prostate cancer [8]. In addition to prostate cancer, changes in CEACAM1 expression and ceACAM1-S/CEACAM1-L ratio promote the growth and metastasis of nonsmall cell lung cancer (NSCLC) [9]. At present, few CEACAM1 related lung cancer studies have been published involving serological studies in patients. Serological diagnosis is convenient, rapid, and noninvasive. If it can be proved that the expression level of CEACAM1 in patients' serum is positively correlated with the poor prognosis of lung cancer patients and can reflect the sensitivity of lung cancer treatment, it will be of great help in clinical work. Therefore, this study aims to find the role of CEACAM1 in the lung cancer signaling pathway through cytological experiments and verify it in serum and tissue samples.

## 2. Data and Methods

### 2.1. General Information

A total of 100 patients with NSCLC who underwent tumor resection and were pathologically diagnosed in the oncology department of Ruijin People's Hospital of Jiangxi Province from March 2013 to March 2018 were screened. Fasting venous blood (5 mL) was collected for each patient before surgery and cancer tissue samples (paraffin sections were prepared) were collected after surgery. In addition, 100 healthy patients without lung cancer who underwent physical examination in our hospital were selected as the control group, and 5 mL venous fasting blood was also collected. Inclusion criteria for study cases: (1) all patients were diagnosed with nonsmall cell lung cancer after pathological diagnosis; (2) the patient's blood routine, coagulation function, and liver and kidney function were normal; (3) the expected survival time is  > 3 months. Exclusion criteria: (1) patients with hemoptysis, hematemesis, and hematochezia; (2) patients with hypertension and uncontrolled proteinuria; (3) patients who have other uncontrollable factors or refuse treatment.

In the patient group, there were 64 males and 36 females, ranging from 30 to 75 years old, with an average age of (56.25 ± 3.52) years old. According to pathological diagnosis, there were 55 adenocarcinoma cases and 47 squamous cell carcinoma cases. Among the healthy subjects, there were 57 males and 43 females, ranging from 31 to 73 years old, with an average age of (55.98 ± 3.39) years old. None of the patients had any diseases other than lung cancer that could affect the results of the analysis. The patients and their families were informed of the details and signed the relevant agreement documents. By comparing the general data such as age and gender, there was no significant difference between the two groups (*P* > 0.05).

The article "Serum Level of CEACAM1 in Patients with Nonsmall Cell Lung Cancer and Its Clinical Significance in Cancer Tissue" was retracted in 2023. Reasons: signs of a paper mill; suspected computer-generated content; unreliable results or conclusions; concerns about the data.

### 2.2. Immunohistochemical Test Method

The cancer tissue was placed in liquid paraffin, and after the paraffin was completely frozen and turned into a solid state, the embedded tissue was placed on a paraffin slicer for sectioning. Tweezers were used to place the slices in warm water at 70°. The slices were removed when fully unfolded and marked. They were placed in the oven to dry for 2 hours.

After sections were dewaxed and washed repeatedly with distilled water, they were soaked in hydrogen peroxide for 10 minutes and then cleaned again. They were placed in a container, citric acid buffer was added, and they were cooked in microwave oven until boiling and cooled for a short time and cooked again for 20 minutes and then cooled to room temperature and antigen sites were exposed. The tissue sections were soaked with phosphoric acid buffer for five minutes, hydrogen peroxide was added to the tissue sections, they were put in a warming chamber for 15 minutes to ensure endogenous oxidase inactivity, they were washed for 2-3 times and then put in the phosphoric acid buffer for cleaning again, serum was dropped to block nonspecific sites, the serum was diluted and 50 ml–100 ml of preprepared primary antibody working solution was added. Primary antibody working solution includes CEACAM1 antibody (AmyJet Scientific), TGF-*β* antibody (ChemicalBook), VEGF-A antibody (Abcam), and IL-8 antibody (Abcam). The control group was replaced by phosphoric acid buffer, placed in the refrigerator of 4°C for 24 hours, and then removed. The second antibody working solution of 50 ml–100 ml was washed with the phosphoric acid buffer for 3 times, 5 minutes each time. The second antibody working solution of 50 ml–100 ml was added, and the second antibody working solution was placed in the incubator for 30 minutes. After rinsing with water, it was placed in hematoxylin for redyeing and then placed successively in alcohol with different concentrations (95%, 85%, 80%, 75%, and 100%) for 2 minutes for each bottle and then soaked in xylene for 2 times for 5 minutes each time, then sealed with neutral gum, dried, and placed under a microscope for observation.

When serum protein was measured, serum cells were isolated and then added to digestive juices for digestion. The cells were suspended using complete culture medium. Cell suspension was added to the cell climbing slice to make the cell patch grow. After the cell growth was stabilized, the slides were added to the stationary liquid for 20 min, and then the confining liquid was dropped for 15 min. Antibody was then dropped onto the slide; the subsequent procedure is the same as that for tissue sample testing.

The article "Serum Level of CEACAM1 in Patients with Nonsmall Cell Lung Cancer and Its Clinical Significance in Cancer Tissue" was retracted in 2023. Reasons: signs of a paper mill; suspected computer-generated content; unreliable results or conclusions; concerns about the data.

### 2.3. Observation Indicators

The evaluation indexes of this study were mainly the detection indexes of CEACAM1, TGF-*β*, VEGF-A, and IL-8 in the serum and tissue samples of patients, and the expression of each indicator and clinicopathological parameters and their correlation were discussed.

### 2.4. Evaluation Criteria

The positive criterion of CEACAM1: the expression of CEACAM1 is mainly presented by staining and divided according to the degree of color development: 0 points (colorless), 1 points (light yellow), 2 points (yellow), and 3 points (brown), among which 0 points and 1 points are negative, and the rest are positive. The field of view is selected under a light microscope, and 500 cells are counted, and the percentage of positive cells is scored. 0 to 5% is negative expression of CEACAM1, and the rest are positive expression.

Positive discriminant criteria for TGF-*β*: after adding the corresponding antibody, a field of 500 cells was selected under a light microscope, and the positive cells were brown or yellow, the proportion of 0 to 20% was negative, and the proportion of more than 20% was positive.

The positive discriminant standard of VEGF-A: after adding the corresponding antibody, the field of vision was selected under the light microscope, with A number of 200 cells. The positive cells were brown or yellow, the negative cells accounted for 0 to 10%, and the positive cells accounted for more than 10%.

Criteria for positive IL-8: after adding the corresponding antibody, the field of vision was selected under a light microscope, and a number of 200 cells were selected. The positive cells were brown or yellow, the negative cells accounted for 0 to 25%, and the positive cells accounted for more than 25%.

### 2.5. Statistical Analysis

Import all collected detection data into SPSS20.0 software for processing and analysis. Measurement data were expressed as mean ± standard deviation (*x* ± *s*), and counting data were expressed as probability %. *T* test was used for comparison between the two groups, and *χ*^2^ test was used for comparison between multiple groups. If *P* < 0.05, it was proved that the difference was statistically significant.

## 3. Results

### 3.1. Comparison of Serum Indicators between NSCLC Patients and Healthy Subjects

After data statistics, it was found that the results of serum indexes in lung cancer group were much higher than that in healthy group (*P* < 0.05). See Table 1 for detailed data.

The article "Serum Level of CEACAM1 in Patients with Nonsmall Cell Lung Cancer and Its Clinical Significance in Cancer Tissue" was retracted in 2023. Reasons: signs of a paper mill; suspected computer-generated content; unreliable results or conclusions; concerns about the data.

### 3.2. Comparison between the Expression of CEACAM1 and TGF-*β* in Cancer Tissues and Clinicopathological Features

The expressions of CEACAM1 and TGF-*β* were correlated with clinical differentiation level, lymph node metastasis, and stage (*P* < 0.05), but were not correlated with gender, age, and tumor diameter (*P* > 0.05). Detailed data are shown in Table 2.

### 3.3. Correlation between CEACAM1 and TGF-*β* Protein Expression in Cancer Tissue

The results of both CEACAM1 and TGF-*β* in cancer tissues were positive in 53 patients and negative in 17 patients, with a consistent rate of 70% (70/100). There was a significant positive correlation between the expression of CEACAM1 and TGF-*β*, which proved that CEACAM1 and TGF-*β* played a synergistic role in the development of NSCLC. See Table 3 for detailed data.

### 3.4. Comparison of the Relationship between the Expression Pattern of CEACAM1 in Adenocarcinoma and Squamous Cell Carcinoma Tissues and Clinicopathological Features of Patients

According to statistical analysis of the data, it was found that the later the clinical stage and the higher the differentiation degree of the cancer tissue specimens of the patients, the more the CEACAM1 expression pattern in the serum samples was expressed in the cytoplasm (*P* < 0.05). Detailed data are shown in Table 4.

## 4. Discussion

Lung cancer is the most dangerous among the common malignant tumors in China and causes the most deaths of all cancers each year [10]. At present, the main clinical treatment means are tumor resection and postoperative chemotherapy. Although medical technology has matured in recent years, the problem of tumor proliferation and implantation is still inevitable, and the therapeutic effect has not reached the expected level. For this reason, it is of certain practical significance to explore the mechanism of the formation and development of lung cancer and provide new targets for clinical examination and future targeted therapy of lung cancer patients.

Human carcinoembryonic antigen associated cell adhesion molecule 1 (CEACAMl) belongs to the carcinoembryonic antigen immune superfamily. Its biological functions include promoting the generation of blood vessels and lymphatics, immunomodulatory regulation of cell proliferation and apoptosis [11], and other pathological processes [7]. Transforming growth factor-*β* (TGF-*β*) is a multifunctional polypeptide cytokine, which is responsible for regulating cell growth and differentiation, apoptosis, angiogenesis, and cellular immunity [12]. TGF-*β* can stimulate tumor cell angiogenesis, which overlaps with CEACAM1. Studies have proved that TGF-*β* can promote the body's autoimmune system by regulating CEACAM1 and play a role in the treatment of systemic lupus erythematosus. We wanted to show whether there was a regulatory relationship between the two in the progression of lung cancer.

The article "Serum Level of CEACAM1 in Patients with Nonsmall Cell Lung Cancer and Its Clinical Significance in Cancer Tissue" was retracted in 2023. Reasons: signs of a paper mill; suspected computer-generated content; unreliable results or conclusions; concerns about the data.

VEGF-A, a member of the VEGF family, is a tumor growth factor that promotes blood vessel growth [13], It plays an important role in tumor angiogenesis by promoting vascular proliferation and division after binding to the receptor. Interleukin (IL-8) is a chemokine in the neutrophil region, which promotes division of proto-activated protein kinases and ultimately tumor development [11].

This study analyzed the expression of CEACAM1 in serum of patients with nonsmall cell lung cancer. The serum index of lung cancer group was higher than that of healthy group. The expression of CEACAM1 and TGF-*β* was correlated with the level of clinical differentiation, lymph node metastasis, and stage, but not with gender, age, and tumor diameter. CEACAM1 was positively correlated with TGF-*β* expression. These results suggest that CEACAM1 and TGF-*β* have synergistic effect on the development of NSCLC. These results indicate that CEACAM1 is sufficient to become an important indicator for the clinical diagnosis of lung cancer patients and provide a target for future targeted therapy of lung cancer. In this study, the expression of CEACAM1 and TGF-*β* and the pathological parameters of lung cancer were further analyzed, and the results showed that the expression of CEACAM1 in lung cancer was roughly divided into three types, namely, cell membrane, cytoplasm, and mixed expression. In addition, the later the clinical stage and the higher the degree of differentiation, the more the cytoplasmic expression of CEACAM1, which provides a theoretical basis for the early diagnosis and clinical treatment of lung cancer. In future related studies, CEACAM1 can be used to regulate lung cancer tumor, and the expression level of CEACAM1 can be used as the criteria for early diagnosis and the basis for middle and late treatment of lung cancer [14, 15].

At present, this experiment has some limitations. The methods for first detection of protein expression are lack of diversity and persuasive. Secondly, the correlation between CEACAM1 in NSCLC tissues and known gene mutations such as EGFR, ALK, and Her2 has not been investigated in depth. In future related studies, the form should be further expanded to ensure the authenticity and effectiveness of research data. In conclusion, serum CEACAM1 levels in patients with NSCLC were not significantly associated with the patient's general data and were significantly increased compared with healthy subjects. In addition, the expression level of CEACAM1 in the serum of NSCLC patients is strongly correlated with TGF-*β*, VEGF-A, and IL-8 in tissue specimens, indicating that the expression of CEACAM1 plays a crucial role in the formation and development of NSCLC. It also proved that serum levels of CEACAM1 and TGF-*β* could predict the occurrence, progression, and outcome of lung cancer, which provides a target for future targeted therapy of lung cancer. Whether the expression of CEACAM1 and TGF-*β* is correlated in lung cancer and whether the two can synergistically participate in the occurrence and regulation of lung cancer can be the focus of future research.

The article "Serum Level of CEACAM1 in Patients with Nonsmall Cell Lung Cancer and Its Clinical Significance in Cancer Tissue" was retracted in 2023. Reasons: signs of a paper mill; suspected computer-generated content; unreliable results or conclusions; concerns about the data.

## Figures and Tables

**Table 1:** Comparison of serum indicators between NSCLC patients and healthy subjects (*X* ± *S*).

Group	Cases	CEACAM1 (ng/mL)	TGF-*β* (ng/mL)	VEGF-A (ng/mL)	IL-8 (ng/mL)
NSCLC groups	100	37.9 ± 14.1	31.7 ± 12.6	553.5 ± 165.6	1.5 ± 0.6
Health groups	100	0.6 ± 0.2	10.7 ± 10.8	116.7 ± 20.8	0.4 ± 0.1
*t*		9.47	7.67	14.10	12.41
*P* value		≤0.001	≤0.001	≤0.001	≤0.001

**Table 2:** Relationship between the expression of CEACAM1 and TGF-*β* in cancer tissues and clinicopathologic features (*n* (%)).

Clinicopathologic parameters		Cases	Relative expression of CEACAM1			Relative expression of TGF-*β*		
			Positive	*χ* ^2^	*P* value	Positive	*χ* ^2^	*P* value
Gender	Male	64	40(62.5)	1.105	0.552	46(71.8)	1.542	0.493
	Female	36	23(63.9)			25(69.4)		
Age (years)	≥60	45	30(66.7)	1.455	0.255	33(73.3)	1.176	0.301
	<60	55	31(56.4)			37(67.2)		
Tumor diameter (cm)	<3	41	24(58.5)	1.071	0.769	27(65.8)	2.947	0.804
	≥3	59	38(64.4)			44(74.6)		
Tumor types	Adenocarcinoma	55	34(61.8)	1.258	0.212	39(70.9)	7.258	0.189
	Squamous cell carcinomas	47	40(85.1)			42(89.4)		
Lymph node metastasis	Yes	45	34(75.6)	6.463	≤0.001	37(82.2)	6.281	≤0.001
	No	35	8(24)			13(37.1)		
Clinical staging	I, II	43	20(47)	5.179	0.022	25(58.1)	7.817	≤0.001
	III, IV	57	47(82)			51(89.5)		
The degree of differentiation	Low/medium	66	57(86.4)	10.847	≤0.001	60(90.9)	8.650	≤0.001
	High	34	17(50)			21(61.8)		

**Table 3:** Relationship between CEACAM1 and TGF-*β* protein expression (*n* (%)).

CEACAM1	TGF-*β*	
	Positive	Negative
Positive	53	10
Negative	20	17

**Table 4:** Relationship between the expression of CEACAM1 and TGF-*β* in cancer tissues and clinicopathologic features (*n* (%)).

Clinical pathological parameters		Cases	CEACAM1 expression pattern				
			Expression in cell membrane	Expression in cytoplasm	Mixed expression	*χ* ^2^	*P* value
Tissue type	Squamous cell carcinoma tissue	55	27(49.1)	14(25.5)	14(25.5)	11.519	0.003
	Adenocarcinoma	47	8(17.0)	28(59.6)	11(23.4)		
The degree of differentiation	Low/medium	66	6(9.1)	35(53.0)	25(37.9)	12.176	0.016
	High	34	12(35.3)	12(35.3)	10(29.4)		
Clinical stage	I, II	43	10(23.3)	23(53.5)	10(23.3)	2.149	0.002
	III, IV	57	6(10.5)	37(64.9)	14(24.6)		

The article "Serum Level of CEACAM1 in Patients with Nonsmall Cell Lung Cancer and Its Clinical Significance in Cancer Tissue" was retracted in 2023. Reasons: signs of a paper mill; suspected computer-generated content; unreliable results or conclusions; concerns about the data.

## Data Availability

The data that support the findings of this study are available on request from the author. The data are not publicly available because they contain information that could compromise research participant privacy.

## References

[1] Ferlay J., Soerjomataram I., Dikshit R. (2015). Cancer incidence and mortality worldwide: sources, methods and major patterns in GLOBOCAN 2012. *International Journal of Cancer*.

[2] Thawani R., McLane M., Beig N. (2018). Radiomics and radiogenomics in lung cancer: a review for the clinician. *Lung Cancer*.

[3] Kim E. S. (2016). Chemotherapy resistance in lung cancer. *Lung Cancer and Personalized Medicine*.

[4] Jacobsen M. M., Silverstein S. C., Quinn M. (2017). Timeliness of access to lung cancer diagnosis and treatment: a scoping literature review. *Lung Cancer*.

[5] Ruiz-Bañobre J., Pérez-Pampín E., García-González J. (2017). Development of psoriatic arthritis during nivolumab therapy for metastatic non-small cell lung cancer, clinical outcome analysis and review of the literature. *Lung Cancer*.

[6] Hasan N., Kumar R., Kavuru M. S. (2014). “Lung cancer screening beyond low-dose computed tomography: the role of novel biomarkers. *Lung*.

[7] Kim W. M., Huang Y.-H., Gandhi A., Blumberg R. S. (2019). CEACAM1 structure and function in immunity and its therapeutic implications. *Seminars in Immunology*.

[8] Qian W., Huang P., Liang X., Chen Y., Guan B. (2020). High expression of carcinoembryonic antigen-associated cell adhesion molecule 1 is associated with microangiogenesis in esophageal squamous cell carcinoma. *Translational Cancer Research*.

[9] MacDonagh L., Gray S. G., Breen E. (2016). Lung cancer stem cells: the root of resistance. *Cancer Letters*.

[10] Torre L. A., Siegel R. L., Jemal A. (2016). Lung cancer statistics. *Lung Cancer and Personalized Medicine*.

[11] Long L., Zhao C., Ozarina M., Zhao X., Yang J., Chen H. (2019). Targeting immune checkpoints in lung cancer: current landscape and future prospects. *Clinical Drug Investigation*.

[12] Soo R. A., Lim S. M., Syn N. L. (2018). Immune checkpoint inhibitors in epidermal growth factor receptor mutant non-small cell lung cancer: current controversies and future directions. *Lung Cancer*.

[13] Frezzetti D., Gallo M., Maiello M. R. (2017). VEGF as a potential target in lung cancer. *Expert Opinion on Therapeutic Targets*.

The article "Serum Level of CEACAM1 in Patients with Nonsmall Cell Lung Cancer and Its Clinical Significance in Cancer Tissue" was retracted in 2023. Reasons: signs of a paper mill; suspected computer-generated content; unreliable results or conclusions; concerns about the data.

[14] Zhang L., Yu H., Li D., Qian H., Chen Y. (2021). Spermatorrhea in a Chinese patient with temporal lobe epilepsy: a case report. *Journal of International Medical Research*.

[15] Park J. T., Fernandez Baca Vaca G., Tangen R., Miller J. (2018). Hippocampal transection for stereo-electroencephalography-proven dominant mesial temporal lobe epilepsy in a child: a detailed case report and critical review. *Journal of Neurosurgery. Pediatrics*.

